RETRACTED

# The Value of MRI Combined with AFP, AFP-L3, GP73, and DCP in the Diagnosis of Early Primary Liver Cancer

**DOI:** 10.1155/2022/8640999

**Published:** 2022-10-13

**Authors:** Zhongjing Kang, Kai Jin, Junpeng Jing

**Affiliations:** ^1^Department of Radiology, Songshan General Hospital, Yubei District, Chongqing, China; ^2^Department of Surgical Intensive Care Unit, Huadong Hospital Affiliated to Fudan University, Shanghai, China; ^3^The People's Hospital of Guangxi Zhuang Autonomous Region, Joint inspection center of precision medicine, No. 6 Taoyuan Road, Qingxiu District, Nanning City, Guangxi, China

## Abstract

**Objective:**

To investigate the diagnostic value of magnetic resonance imaging (MRI) combined with serum alpha-fetoprotein (AFP), alpha-fetoprotein (AFP-L3), Golgi protein 73 (GP73), and des-*γ*-carboxyprothrombin (DCP) on early-stage primary liver cancer (PHC).

**Methods:**

A total of 122 patients who were treated in our hospital from January 2019 to May 2022 were included in this study, including 62 patients with early PHC (referred to as the observation group) and 60 patients with benign liver disease (referred to as the control group). MRI scans were performed on all participants, and MRI image features were compared. Subsequently, the differences in serum AFP, AFP-L3, GP73, and DCP concentrations of the two groups of patients were detected and compared. Receiver operating characteristic (ROC) curve was used to analyze the efficacy of MRI and each of the above tumor markers in diagnosing early PHC.

**Results:**

The proportion of low or slightly low signal on T1WI in the observation group was significantly greater than that in the control group, while the proportions of equisignal and high signal were lower than those in the control group. The proportion of high signal on T2WI and high signal on DWI in the observation group was higher than that in the control group, while the proportion of low or slightly low signal and equisignal was lower than that in the control group. Compared with the control group, the serum concentrations of AFP, AFP-L3, GP73, and DCP in the observation group were significantly increased (all *P* < 0.05). For the diagnosis of early-stage PHC patients, MRI combined with these four markers showed favorable diagnostic value compared with parameter alone (area under the ROC curve, sensitivity, and specificity were 0.943, 0.919, and 0.833, respectively).

**Conclusion:**

MRI combined with serum AFP, AFP-L3, GP73, and DCP detection has good value in the diagnosis of early PHC patients, and can serve as an effective strategy to improve the early diagnosis rate of PHC.

## 1. Introduction

Primary hepatic carcinoma (PHC) has a high morbidity and mortality worldwide [1, 2]. Its insidious onset, rapid disease progression, and delayed diagnosis render a missed time for surgical intervention [3, 4]. Therefore, early and accurate diagnosis of PHC is crucial for improving the prognosis of PHC patients. With the rapid progress of diagnostic equipment and diagnostic technology, imaging examinations play an important role in the diagnosis of PHC, among which magnetic resonance imaging (MRI) features multi-sequence, multi-parameter, and multi-directional imaging, and it has been widely used in the diagnosis of PHC [5–8].

RETRACTED

Serum tumor markers also play a very critical role in the diagnosis of tumors. Alpha-fetoprotein (AFP), as a glycoprotein, is a commonly used and highly specific tumor marker for the diagnosis of PHC in clinical practice [9–11]. AFP also has value in the early diagnosis of PHC. Kong et al. reported that the combined detection of enhanced CT and contrast-enhanced ultrasound with tumor markers such as AFP is helpful for the early diagnosis of PHC (35237392). Alpha-fetoprotein-L3 (AFP-L3), a subtype of AFP, has been reported to have high specificity for early PHC diagnosis [12, 13]. In recent years, Golgi protein 73 (GP73) was found to be significantly elevated in the serum of PHC patients, and it was considered a biomarker for diagnosing early PHC [14, 15](33343966). De-*γ*-carboxyprothrombin (DCP) also showed good diagnostic performance for early PHC [16]. In the study of early gastric cancer diagnosis, the combined diagnostic performance of MRI-DWI signal intensity value and serum indicators such as CA199 is better than the diagnostic performance of indicators alone [17].

However, the value of MRI combined with serum tumor markers AFP, AFP-L3, GP73, and DCP in the diagnosis of early PHC has not been explored. Therefore, this study investigated the diagnostic value of MRI combined with these four serum tumor markers for early primary liver cancer, with an aim to provide a reference for the early diagnosis of primary liver cancer.

## 2. Materials and Methods

### 2.1. Baseline Data

A total of 122 patients who were treated in our hospital from January 2019 to May 2022 were included in this study, including 62 patients with early PHC (referred to as the observation group, 35 males and 27 females, aged 26-81 years old, with an average age of 58.56 ± 9.89 years) and 60 patients with benign liver disease (referred to as the control group, 39 males and 21 females, aged 25-82 years, with an average age of 58.45 ± 10.01 years). According to TNM staging, the observation group included 35 patients with stage I and 27 patients with stage II. The baseline data such as age and gender in the two groups of participants were statistically insignificant (*P* > 0.05).

RETRACTED

Inclusion criteria: (1) all PHC patients met the diagnostic criteria for primary liver cancer; (2) all patients were diagnosed by pathology; (3) patients aged 20 to 85 years; (4) complete clinical imaging data. Exclusion criteria: (1) patients who received relevant anti-tumor interventions before admission; (2) patients with other primary malignant tumors; (3) patients with metastatic liver cancer; (4) patients with mental disorders. This study was approved by the hospital ethics committee (No. 2019022), and all participants signed a written informed consent.

### 2.2. Methods

#### 2.2.1. Magnetic Resonance Imaging (MRI)

Scanning of the patient's liver area was done with a GE HDxt3.0 MRI scanner and an 8-channel body phased array coil. Scan sequences included T1-weighted imaging (T1WI), T2-weighted imaging (T2WI), and diffusion-weighted imaging (DWI).

Relevant parameter settings for T1WI: repetition time (TR) is 440 ms, echo time (TE) is 191 ms, slice thickness is 8 mm, slice spacing is 2 mm, field of view (FOV) is 360 mm ×270 mm, matrix is 190 × 120, and the number of excitations (NEX) is 3 times.

Relevant parameter settings of T2WI: TR is 8571 ms, TE is 1916 ms, slice thickness is 6.5 mm, slice spacing is 2 mm, FOV is 350 mm ×350 mm, matrix is 128 × 256, and the number of excitations is 3 times. DWI-related parameter settings: TR is 3200 ms, TE is 94 ms, FOV is 350 mm ×350 mm, matrix is 128 × 128, and NEX is 3 times.

After the routine scan was completed, 15 mL of contrast agent was injected through the cubital vein. After injection, the arterial phase scan was performed at 25 s, the venous phase scan was performed at 60s, and the delayed phase scan was performed at 200 s. Relevant parameter settings: TR is 1200 ms, TE is 78.9 ms, layer thickness is 5 mm, layer spacing is 2 mm, FOV is 400 mm ×400 mm, matrix is 128 × 128, NEX is 1 time, and the *b* value is 500 s/mm2. Finally, the obtained scan data is analyzed by the processing system, and the characteristics such as the shape of the lesion and the signal intensity are observed. The analysis of these data was done on a double-blind basis by two senior radiologists. When the results are inconsistent, the two would decide after joint discussion.

#### 2.2.2. Detection of Serum Tumor Marker Levels

5 mL of fasting cubital venous blood was collected from all subjects before treatment in the morning, and they were left standing at room temperature for 30 minutes before centrifugation (3500 r/min); the serum was obtained and sent for inspection. AFP and AFP-L3 were detected by electrochemiluminescence immunoassay, and the kits were purchased from Wuhan Yipu Biotechnology Co., Ltd.; GP73 and DCP were detected by enzyme-linked immunosorbent assay, and the kits were purchased from Shanghai Luzhen Biotechnology Co., Ltd. and Shanghai Jianglai Biotechnology Co., Ltd., respectively. All operations were carried out in accordance with the kit instructions.

RETRACTED

### 2.3. Outcomes

The MRI image characteristics of the two groups were compared, and the concentrations of serum markers AFP, AFP-L3, GP73, and DCP were compared between the two groups; the area under the ROC curve (AUC), sensitivity, specificity, etc. were calculated, and the ROC curve was drawn and analyzed. The diagnostic value of MRI scan combined with these four serum tumor markers in early PHC was analyzed.

### 2.4. Judgment Criteria

The positive reference values of serum tumor markers AFP, AFP-L3, GP73, and DCP: AFP>400 ng/mL, AFP-L3>40.00 ng/mL, GP73>100 ng/mL, DCP> 40 mAU/ml. A test result below the positive reference values is considered negative.

### 2.5. Statistical Analysis

SPSS 25.0 software was used to analyze data. For enumeration data, chi-square test was used; for quantitative data, the independent samples *t* test was employed. ROC curve analysis was performed using GraphPad Prism 9 and R v.4.2.0, respectively. *P* values of 0.05 or lower were considered to be statistically significant.

## 3. Results

### 3.1. Comparison of Two Groups of MRI Image Features

It can be seen from Table 1 that on T1WI, the proportion of low or slightly low signal in the observation group (PHC group) was significantly greater than that in the control group, while the proportion of equisignal and high signal in the control group was greater than that in the observation group. The proportion of people with high signal on T2WI and high signal on DWI in the observation group were higher than those in the control group, while the proportion of people with low or slightly low signal and equisignal were lower than those in the control group.

### 3.2. Comparison of Serum AFP, AFP-L3, GP73, and DCP Concentrations between the Two Groups

As shown in Table 2, the serum AFP, AFP-L3, GP73, and DCP concentrations in the observation group were higher than those in the control group (all *P* values < 0.05).

### 3.3. Diagnostic Efficacy of Different Diagnostic Methods for Early PHC

According to Table 3 and Figure 1, the AUC value, sensitivity, and specificity of serum tumor markers AFP, AFP-L3, GP73, and DCP combined with MRI in the diagnosis of early PHC were 0.943, 0.919, and 0.833, respectively. The AUC value and sensitivity of the combined diagnosis were higher than those of the individual diagnosis. However, the specificity of the combined diagnosis was 0.833 lower than 0.900 for AFP and 0.850 for AFP-L3.

RETRACTED

## 4. Discussion

PHC is the most common digestive malignancy causing cancer-related deaths in the world, with approximately 780,000 deaths in 2018 alone [1, 18]. At present, its pathogenesis has not been fully elucidated, and it may be related to factors such as genetics, diet, and environment [19, 20]. PHC patients often lack typical symptoms in the early stage, and most of the patients come to the hospital due to symptoms such as jaundice and liver pain. By that time, most of them are already in the advanced stage and lose the best time for radical surgery, resulting in poor prognosis of patients [3, 4, 21]. Therefore, in order to improve the prognosis of patients, early diagnosis of PHC is of great significance. At present, the gold standard for the diagnosis of PHC is still pathological examination; however, its operation will cause damage to patients. MRI scan is helpful to detect lesions in time, but it may be missed and misdiagnosed, so the combined diagnosis with other examination methods may improve the diagnostic performance of PHC. As an important tumor detection method, tumor markers have been widely studied and applied in tumor diagnosis. It has been reported that serum tumor markers AFP, AFP-L3, GP73, and DCP are all valuable for the early diagnosis of PHC, but their diagnostic performance alone is not satisfactory [22–25]. Therefore, it is meaningful to explore the combination of MRI and the above tumor markers to improve the early diagnosis rate of PHC patients.

The results of this study showed that the number of people with low or slightly low signal on T1WI in the observation group (PHC group) was more than the number in the control group, and the number of people with high signal on T2WI and DWI in the PHC group was more than the number in the control group, which is consistent with Yuan et al. studies [26]. The above results suggest that there are differences in T1WI, T2WI, and DWI signals between patients with early PHC and patients with benign liver disease, and these differences can help to determine the nature of the disease. In addition, We found that serum AFP, AFP-L3, GP73, and DCP concentrations were significantly increased in PHC patients in the observation group compared with the control group (all *P* values < 0.05). The reason is that AFP is a glycoprotein mainly synthesized in the embryonic period. For normal adults, its content is very low, while the elevation is mainly seen in patients with liver cancer. At present, it is generally considered to be a marker that can be used for early diagnosis of PHC [27]. AFP-L3 is a PHC-specific marker, mainly secreted by hepatoma cells and able to enter the blood circulation [12]. GP73 is a Golgi type II transmembrane protein, and several researchers have pointed out that its concentration in the serum of PHC patients is increased [14, 23, 28]. When liver cancer occurs, its cells cannot make good use of vitamin K, resulting in a decrease in the activity of vitamin K-dependent *γ*-glutamyl carboxylase and a decrease in the carboxylation of prothrombin precursor, thereby causing a large amount of DCP to be produced and secreted into the blood circulation [29].

RETRACTED

Moreover, this study also analyzed and compared the performance of different examination methods in the diagnosis of early PHC. The AUC value, sensitivity, and specificity of AFP, AFP-L3, GP73, and DCP combined with MRI in the diagnosis of early PHC were 0.943, 0.919, and 0.833, respectively. Among them, the AUC value and sensitivity of the combined diagnosis of serum tumor markers and MRI were higher than those of single diagnosis. The specificity of the combined diagnosis was 0.833, which was lower than 0.900 for AFP and 0.850 for AFP-L3. Overall, the combined diagnosis performed better. This suggests that the combined diagnosis of multiple inspection methods has a certain complementary effect, and the combined diagnosis is helpful to improve the early diagnosis rate of PHC. Therefore, the combination of MRI and serum tumor markers can be considered in clinical diagnosis of PHC to improve the early diagnosis rate of PHC.

## 5. Conclusion

Overall, the combined diagnostic performance of MRI and serum AFP, AFP-L3, GP73, and DCP was superior to each individual diagnostic performance. MRI examination combined with serum AFP, AFP-L3, GP73, and DCP detection may be a useful method for early diagnosis of PHC, and it is worthy of clinical application.

## Figures and Tables

**Figure 1:** ROC curves for each diagnostic modality. (a) ROC curve of a single index. (b) ROC curve of 4 tumor markers combined with MRI.

**Table 1:** Comparison of MRI image features between observation group and control group [*n* (%)].

Test sequence/number	Observation group	Control group
T1WI		
Low or slightly low signal	56 (90.32)	33 (55.00)
Equisignal	2 (3.23)	11 (18.33)
High signal	4 (6.45)	16 (26.67)
T2WI		
Low or slightly low signal	0 (0.00)	5 (8.33)
Equisignal	3 (4.84)	13 (21.67)
High signal	59 (95.16)	42 (70.00)
DWI		
Low or slightly low signal	0 (0.00)	4 (6.67)
Equisignal	0 (0.00)	9 (15.00)
High signal	62 (100.00)	47 (78.33)
N	62	60

**Table 2:** Comparison of serum AFP, AFP-L3, GP73, and DCP concentrations between the two groups (mean ± standard deviation).

Groups	*n*	AFP (ng/mL)	AFP-L3 (ng/mL)	GP73 (ng/mL)	DCP (mAU/mL)
Observation group	62	541.62 ± 46.80	102.80 ± 58.30	134.99 ± 46.31	187.67 ± 54.86
Control group	60	53.60 ± 24.79	26.22 ± 41.38	64.25 ± 24.13	27.68 ± 8.79
t		71.627	8.342	10.530	22.311
*P*		0.021	0.001	≤0.001	≤0.001

RETRACTED

**Table 3:** Efficacy of different diagnostic modalities in the diagnosis of early PHC.

Diagnostic methods	AUC	95% CI	Sensitivity	Specificity	Youden index
AFP	0.695	0.600-0.791	0.581	0.900	0.481
AFP-L3	0.737	0.650-0.824	0.565	0.850	0.415
GP73	0.754	0.667-0.842	0.716	0.800	0.516
DCP	0.750	0.662-0.838	0.867	0.645	0.512
MRI	0.782	0.700-0.863	0.767	0.758	0.525
4 markers + MRI	0.943	0.906-0.981	0.919	0.833	0.752

## Data Availability

No data were used to support this study.
